# Data Mining and Meta-Analysis of Psoriasis Based on Association Rules

**DOI:** 10.1155/2022/9188553

**Published:** 2022-01-27

**Authors:** Jiarui Ou, Jianglin Zhang

**Affiliations:** ^1^Department of Detmatology Xiangya Hospital, Central South University, Changsha, Hunan 410008, China; ^2^Department of Detmatology, Shenzhen People's Hospital (The Second Clinical Medical College,Jinan University; The First Affiliated Hospital,Southern University of Science and Technology), Shenzhen, Guangdong 518020, China

## Abstract

Psoriasis is a common chronic and recurrent disease in dermatology, which has a great impact on the physical and mental health of patients. Meta-analysis can evaluate the effectiveness and safety of defubao in the treatment of psoriasis vulgaris. This article observes psoriasis skin lesions treated with topical defubao and the changes in blood vessels under dermoscopy. Considering that the Apriori algorithm and the existing improved algorithm have the problems of ignoring the weight and repeatedly scanning the database, this paper proposes a matrix association rule method based on random forest weighting. This method uses the random forest algorithm to assign weights to each item in the data set, and introduces matrix theory to convert the transaction data set into a matrix form and store it, thereby improving operating efficiency. This article included 11 studies, of which 7 studies used the indicator “Researcher's Overall Assessment” (IGA) to evaluate the efficacy, 5 studies used the “Patient Overall Assessment” (PGA) as the efficacy evaluation index, and Loss Area and Severity Index (PASI) was used as an observation index to evaluate the efficacy. Seven studies conducted safety comparisons. In this paper, IGA and PGA were used as evaluation indicators. The treatment effect of the defubao group was better than the calcipotriol group and the betamethasone group. The differences were statistically significant. The effect of the Fubao treatment for 8 weeks is significantly better than that of 4 weeks and 2 weeks, and the differences are statistically different. Using PASI as the evaluation index, a descriptive study was carried out, and it was found that after 4 weeks of treatment for psoriasis vulgaris, the average PASI reduction rate of patients was higher than that of the calcipotriol group and the betamethasone group. The safety evaluation found that after 8 weeks of treatment, the incidence of adverse events in the defubao group was significantly lower than that in the calcipotriol group.

## 1. Introduction

How to discover these hidden and valuable relationships has always been a research hotspot in the field of data mining [1, 2]. Among them, data mining technology refers to a large number of data sets, through association rule mining, classification, aggregation and outlier detection and other methods, to find the internal relationship between the data in the data set without obvious characteristics, so as to guide people in subsequent production activities. For example, in the typical case of retail data on beer and diapers, if the decision-makers did not use data mining technology to effectively analyze the retail data, how could they find that people who bought beer would also buy diapers? Among them, in the case of beer and diapers, association rules technology is used, which is a very practical data mining technology [3–5]. This mining technology has been widely used in many fields such as store layout, consumer behavior, accident data analysis, and fraud detection [6, 7].

Psoriasis, known as “white boil” in traditional Chinese medicine, is a common chronic, inflammatory, and recurrent skin disease [8]. It is characterized by red papules or plaques with multiple layers of silvery white scales covering the limbs. Extensive side, scalp and back, severe skin lesions can spread all over the body, accompanied by varying degrees of itching [9, 10]. The disease can be seen in all races, and the prevalence varies among different regions and races. Psoriasis is clinically divided into 4 types, including vulgaris, erythroderma, pustular, and articular types, among which vulgaris is the most common, accounting for more than 97% of all patients [11]. Common TCM syndrome differentiation mainly includes blood syndrome, blood heat syndrome, blood dryness syndrome, blood deficiency syndrome and blood stasis syndrome [12]. However, psoriasis persists for a long time and the pathogenesis is complicated. Only four types cannot meet the complex and changeable clinical syndrome differentiation needs of psoriasis vulgaris. At present, our country is in a period of social transformation and rapid economic growth, and the subsequent air pollution, water pollution and increasing living pressure have laid hidden dangers for the occurrence of this disease [13]. Therefore, the need for research and treatment of this disease is more urgent than in any previous period. Modern medicine has been continuously exploring and researching the disease, and there have been a lot of research results. However, the etiology and pathogenesis of psoriasis are still unclear. Its treatment has large side effects and lacks safe, effective and satisfactory long-term curative effects. This article aims to systematically collect patients' symptoms, related factors, and analyze the distribution characteristics of pathogenic factors, combination characteristics, distribution of related factors and typical symptoms caused by pathogenic factors as comprehensively as possible, and discuss the differentiation of psoriasis vulgaris [14]. Element characteristics, using the simple, flexible, accurate, and comprehensive characteristics of syndrome elements to describe the pathogenesis of psoriasis vulgaris, provide a basis for more accurate and effective differentiation and treatment of psoriasis vulgaris [15]. In this way, the complex pathogenesis is divided into several syndrome differentiation elements of the combination of syndromes, and the precise differentiation of syndromes can be used to guide the treatment more accurately, so as to be beneficial to more in-depth research on the disease and to further improve the clinical efficacy of the disease. At present, the common indicators for evaluating the severity of psoriasis include skin lesion area and severity index, the researcher's overall assessment, the patient's overall assessment, and the target skin lesion score. The first three indicators are to observe and evaluate the overall severity of the patient. Target lesion scores are widely used to assess the severity of specific lesions in psoriasis. It includes erythema, scale, and infiltration. TLS observes specific local skin lesions. Therefore, when it is necessary to combine auxiliary examination methods to dynamically observe and record changes in diseases or skin lesions, TLS is more intuitive and comparative.

Calcipotriol has been widely used in the treatment of psoriasis, and its efficacy and safety have been recognized by doctors and patients. Local topical glucocorticoids are also the first choice for the treatment of psoriasis. Before the advent of defubao, the effect of using glucocorticoid in the morning and calcipotriol at night was significantly better than using calcipotriol or glucocorticoid alone twice a day. Topical calcipotriol and glucocorticoids have been used as classic first-line drugs for the treatment of psoriasis for several years. Calcipotriol is a vitamin D derivative, which can regulate the proliferation and differentiation of epidermal cells, as well as the production and release of pro-inflammatory cytokines. Local topical glucocorticoid therapy will have a wide range of biological effects, such as inhibiting the production and migration of inflammatory cells, regulating the release of cytokines (such as IL-2) and chemokines, and regulating DNA synthesis. However, external hormones alone have side effects, including skin atrophy, telangiectasia, and uneven pigmentation. Defubao is a compound preparation of betamethasone and calcipotriol, containing calcipotriol 50 *μ*g/g and betamethasone dipropionate 0.5 mg/g. Defubao was approved by the State Food and Drug Administration for the treatment of psoriasis vulgaris. In theory, it has both calcipotriol's pro-keratinocyte differentiation effect and betamethasone anti-inflammatory effect, which combines the advantages of the two drugs and complements the side effects of the two drugs. However, the effectiveness and safety of defubao still need strong evidence-based medical evidence to objectively evaluate.

## 2. Related Work

Many scholars have proposed binding and nonbinding association rules [16–18]. For example, they add restrictions on the number of transactions and transaction time to each item in the database to reduce the number of association rules, generate only interesting rules, generate only nonredundant rules, or use sampling to display association rules, or generate only those that meet certain requirements [19].

Relevant scholars have adopted the maximum utility value strategy, and proposed the LQS-tree storage structure, item connection and sequence connection to expand the sequence, and also provided width pruning and deep pruning to prune undesirable sequences [20]. Related scholars have proposed a four-stage MapReduce framework, which is completely based on the famous Spark platform for mining HUSP [21]. The framework provides more efficient and faster mining performance for processing large data sets. It includes four stages: initialization, mining, update, and generation. It is based on the MapReduce framework running on the Spark platform to process large data sets.

At present, most of the algorithms are mainly focused on HUSP mining in static databases, without considering streaming data. In streaming data, unlimited data appears continuously and at a high speed, which will increase the difficulty of mining. Based on this, related scholars have proposed a HUSP-UT algorithm, which is based on a data stream tree structure [22, 23]. A large number of experiments on real data sets show that HUSP-UT can effectively identify high-efficiency sequences. In addition, the article also proposes a new upper bound-sequence expansion utility. A variety of pruning strategies are further adopted [24].

In the real world, the time interval between elements is also very important. However, the existing HUSP mining algorithms cannot extract sequential patterns of this nature. The researchers took into account the utility of the elements and the time interval, and proposed a sequential pattern mining algorithm with the nature of time interval [25, 26]. In addition, four time constraints are used to process the time intervals in the sequence to extract more meaningful patterns. In addition, two upper bounds of utility are proposed, namely the upper bound of residual utility (RUUB) and the upper bound of co-occurrence utility (CUUB) to prune hopeless candidates. Under the assumption that multiple events can occur simultaneously and persist for different periods of time, considering the utility of events, a pattern mining algorithm based on high-efficiency intervals, HUIPMiner, is proposed [27, 28].

Relevant scholars believe that psoriasis is related to the five internal organs, and is most closely related to the liver [29]. The main factors are that the liver controls drainage, the blood storage in the liver, and the pathological interaction between the liver and other internal organs. Scholars used a multi-center randomized controlled method for clinical observation [30]. The treatment group was mainly given the prescription of cooling blood and detoxification, the liver-clearing and purging gunpowder was used for the blood-heat syndrome, the liver-releasing and qi-regulating medicine was used for the blood stasis syndrome, and the liver-softening detoxification was used for the blood-dry syndrome [31–33]. All were treated with medicine that was soothing to the liver and relieved depression. The improvement of DLQI scores in the treatment group was better than those in the control group. Therefore, the treatment of psoriasis from the liver theory based on Liangxue Jiedu Decoction can effectively improve the degree of skin lesions, TCM syndromes and quality of life [34, 35].

The TCM syndrome differentiation type included in the literature lacks objective and unified standardized standards. The outcome index adopts the comprehensive curative effect evaluation index, and the improvement of symptoms is based on the subjective judgment of the investigator, which makes the judgment of curative effect lack objectivity. In addition, in the trial design, most of the literature lacks long-term follow-up, which affects the combined analysis of the long-term efficacy of external use of traditional Chinese medicine in the treatment of psoriasis vulgaris. This may be related to the long treatment period of traditional Chinese medicine and the relatively difficult follow-up. A small part of the literature even lacks the description of the adverse reaction, and most of the literature lacks objective basis when describing the adverse reaction, which reduces the completeness of the data.

## 3. Method

### 3.1. Mining Based on Apriori Text Association Rules

The following introduces the related concepts of Apriori and the main algorithm process in two parts.

(1) Support: For a given data set, how often certain features are found. Support is defined as follows:
  (1) $$\begin{array}{c} \sup\text{port}\left(A,B\right)=P\left(A\subseteq B\right)\cup P\left(A\cap B\right). \end{array}$$
Among them, A and B are itemsets.
(2) Confidence degree: It reflects the certainty of the reflection rules on the basis of frequent itemsets. The confidence is defined as follows:
  (2) $$\begin{array}{c} \text{Confidence}\left(A,B\right)=P\left(A\cup B\right)\cap P\left(A\cap B\right). \end{array}$$
(3) Frequent itemsets: Frequent itemsets find the set of data that is not less than the minimum support degree.
(4) Strong association rules: On the basis of frequent itemsets, strong association rules also meet artificially set thresholds.

Apriori's algorithm uses the candidate function to generate frequent itemsets. The function first counts the number of occurrences of each element in the itemsets (also known as support count), and finds the frequent itemsets. Then the function rescans the data set, using the iterative layer-by-layer method until there is no maximum itemset generated. The calculation process of Apriori is shown in Figure 1.

### 3.2. Diagnostic Model Construction Method

RNN and DBN can also achieve better experimental results in practical applications. However, these two methods still have problems in processing text data. In view of the shortcomings of the above methods, CNN, as a typical neural network, can solve the above problems well. As a feedforward network, it has outstanding performance in reducing weights and computational complexity.

The input data has a certain format, and the image itself is composed of multiple pixels, so it has certain regularity. For text data, the converted word vector is generally used as input data.

To extract the features of the input data *x*(*i*), the discrete convolution formula is

(3) $$\begin{array}{c} y\left(n\right)=\prod_{i=0}^{\infty }\left[h\left(n-i+1\right)•x\left(i+1\right)\right]. \end{array}$$

Among them, *h*(*n *−* i*) is the convolution kernel.

A filter is also called a convolution kernel. Assuming that the length of the input data is *n* and the size of the convolution kernel is *m*, the feature length after the convolution operation is *n *−* m *+* *1. However, this situation will reduce the length of the feature. CNN adopts an expansion method, that is, filling the boundary of the input data to prevent problems caused by size changes.

The feature matrix obtained by convolution has a relatively large dimension and cannot accurately describe data features. After pooling, more accurate features can be obtained, which is convenient for subsequent work.

TextCNN optimizes the standard CNN convolutional layer structure, which uses simple models to achieve excellent results in multiple data sets, achieves end-to-end classification effects, and makes it better to process text content. Compared with CNN, the network structure is simple, and the input data is one-dimensional data. The biggest feature of TextCNN is to classify text. The data are mapped to a low-dimensional space for encoding through the feature extractor of the embedding layer.  Figure 2 shows the architecture of the psoriasis data mining system based on association rules.

### 3.3. Random Forest Algorithm

The algorithm principle is as follows:

1. The sample is replaced with *n* samples randomly selected as the training set.
2. Use the training set to construct a decision tree, and randomly extract features during the construction process.
3. Repeat the above process to generate multiple decision trees.
4. Integrate all decision trees to predict new data (the majority vote is generally used for classification).

The random forest algorithm can effectively weigh each feature in the data set. The main idea is to calculate the average contribution of each feature in the random forest for all trees in the random forest. The Gini index is commonly used as a measurement indicator. The process of random forest algorithm is shown in Figure 3.

Here, VIM is used for variable importance measures, and *GI* is used for Gini index. Taking a data set containing *n* features as an example, the calculation method of the *j*-th feature Gini index score VIM_*j*_(Gini) is:

(4) $$\begin{array}{c} GI_{m}=\prod_{k=0}^{K}\prod_{k^{\prime }=1}^{K}\left(p_{mk}p_{mk^{\prime }}\right), \end{array}$$

where *K* represents the number of categories included, and *P*_*mk*_ represents the probability of randomly sampling two samples of different categories from node *m*. The importance of feature *X*_*j*_ to node *m* is:

(5) $$\begin{array}{c} {\text{VIM}}_{jm}^{Gini}+GI_{l}=2GI_{r}+GI_{m}. \end{array}$$

Here, *GI*_*l*_ and *GI*_*r*_, respectively, represent the Gini index of the new node after branching. If the node of feature *X*_*j*_ in decision tree *i* belongs to set *M*, then the importance of *X*_*j*_ to the *i*-th tree is:

(6) $$\begin{array}{c} {\text{VIM}}_{ij}^{Gini}=\prod_{m⟶M}\left({\text{VIM}}_{jm}^{Gini}+GI_{l}+GI_{r}+GI_{m}\right),\\ {\text{VIM}}_{j}^{Gini}=\prod_{i=0}^{n-1}\left({\text{VIM}}_{ij}^{Gini}-GI_{l}-GI_{r}-GI_{m}\right). \end{array}$$

### 3.4. Design of Matrix Association Rule Algorithm Based on Random Forest Weight

The traditional Apriori algorithm and the existing improved algorithm have problems such as low operating efficiency, and many redundant rules. In response to these problems, this section combines the random forest algorithm with matrix theory, proposes a matrix association rule algorithm based on random forest weights, and designs and implements related comparative experiments.

Due to the introduction of weights, the traditional support and confidence are no longer applicable. In addition, the transformed matrix needs to be compressed according to related properties to further obtain frequent itemsets. Therefore, this paper defines the weighted support and weighted confidence, and provides related definitions and proofs for matrix compression.

*W*(*X*) is recorded as the weight of item set *X*, which represents the sum of the weights of all items in item set X:

(7) $$\begin{array}{c} W\left(X\right)=\sum_{i,I\left(X\right)}\left[W\left(i_{j}\right)+GI_{l}+GI_{r}+GI_{m}\right]|\prod_{i,I\left(X\right)}W\left(i_{j}\right). \end{array}$$

*W*Sup(*X*) is recorded as the weighted support of item set *X*:

(8) $$\begin{array}{c} W\text{Sup}\left(X\right)=W\left(X\right)•W\left(X\right)•\text{Sup}\left(X\right). \end{array}$$

If *W*Sup(*X*)* *>* *minsup (customized minimum weighted support), then the item set *X* is called a weighted frequent set. The weighted confidence of the association rule *X*-*Y* is:

(9) $$\begin{array}{c} W\text{Conf}\left(X\mapsto Y\right)=W\text{Sup}\left(X\cap Y\right)|W\text{Sup}\left(X\cup Y\right). \end{array}$$

Suppose there is a transaction data set *D* = {*t*1, *t*2, *t*3, *t*4, *t*5}, and its corresponding item set is I = {I1, I2, I3, I4, I5}. First, we scan the transaction data set *D*, and obtain the weight of each feature through the above random forest method. The conversion method is, if the *j*-th item exists in the *i*-th transaction, we set the value of the *i*-th row and the *j*-th column of the matrix to 1, otherwise set its value to 0. The transformed transaction matrix D1 is shown in Table 1.

On the basis of the converted matrix, we add two new rows Sup and WSup, and add a new column sum_c, where sum_c is used to record the total number of items contained in each transaction, and Sup and WSup are used to record the support of different items, respectively.

We set the minimum weighted support min_wsup, compare the support number of each item recorded in the last row, if the support number of an item is not less than min_sup, it will be recorded as frequent 1 item set, otherwise the corresponding column will be deleted. If the value corresponding to an element is 0, we delete the corresponding row to obtain a new transaction matrix.

This process is repeated all the time, resulting in frequent *k* itemsets (*k* ≥ 2). We delete the matrix column corresponding to the item Ij that appears less than *k* in the frequent *k *−* *1 item set and recalculate the sum_c column of the matrix. According to property 2, if the value of an element is less than *k*, we delete the corresponding row of the element in the matrix. If the value of an element is less than min_sup, we delete the column corresponding to the element.

### 3.5. Statistical Processing

RevMan 5.3 software was used for meta-analysis of the data. First, X2 is used to evaluate the heterogeneity between similar studies. If *P* ≥ 0.1 and I2* *≤* *50%, it means that there is homogeneity between the studies, and the fixed effects model is used for meta-analysis; if *P* < 0.05, I2* *>* *75%, it is considered that there is heterogeneity between the studies and the heterogeneity should be analyzed. After subgroup analysis is conducted according to the research design and different treatment options, and after eliminating the problems of the quality of the research design and different treatment options, the random effects model can be used to combine the effect size, and the research results can be explained carefully. Sensitivity analysis is performed on the heterogeneity caused by different research methods, and different model calculations are performed to evaluate the stability of the meta-analysis results. The outcome variables of this study are all two-category count data, and the odds ratio and 95% confidence interval are used as the analysis statistics. For those with insufficient data in clinical trials, only descriptive analysis will be performed.

## 4. Results and Discussion

### 4.1. Effectiveness Analysis

There are 4 randomized trials to evaluate and compare the effectiveness of defubao and betamethasone in the treatment of psoriasis vulgaris through IGA indicators. According to the course of treatment, they are divided into 3 subgroups: treatment for 2 weeks, treatment for 4 weeks, and treatment for 8 weeks. After 2, 4, and 8 weeks of treatment, the proportion of patients in the defubao group whose IGA assessment changed to “regression of skin lesions” or “very mild skin lesions” was significantly higher than that of the betamethasone group. The group had no heterogeneity in each outcome index, so fixed effects models were used for meta-analysis. The results showed that whether the treatment course was 2 weeks or 8 weeks, the treatment effect of defubao was significantly better than that of betamethasone, and the difference was statistically significant. The IGA used the IGA as an indicator to evaluate the asymmetry of the funnel chart between the defubao group and the betamethasone group at 8 weeks, and there is a publication offset in the study, as shown in Figure 4. However, in the subgroup comparing the efficacy of 4 weeks, the Cochrane *Q* analysis suggests that the combined data of the three groups are significantly heterogeneous, so the 4-week period is valid. The conclusions reached suggest that after 4 weeks of treatment, the treatment effect of the defubao group is better than that of the betamethasone group.

Three trials compared the effectiveness of defubao and calcipotriol (1* *time/day) using IGA as an observation indicator. According to the different treatment time, they are divided into 3 subgroups and compared separately. The difference in curative effect of treatment for 2 weeks, treatment for 4 weeks, and treatment for 8 weeks is mainly compared. The 2-week curative effect subgroup and the 8-week curative effect subgroup, respectively. A fixed effects model was used for data analysis. As shown in Figure 5, the funnel graph is asymmetric, and the research has a publication offset. There is significant heterogeneity in the three groups of data compared between the four-week efficacy subgroups, and the random effects model is selected for data analysis. The results showed that the treatment with defubao was applied in 2 weeks [OR = 5.49, 95%CI (4.27, 7.05), *P* < 0.001], 4 weeks [OR = 4.67, 95%CI (3.31, 6.57), *P* < 0.001], and 8 weeks [OR = 3.44, 95% CI (2.78, 4.25), *P* < 0.001], and the effective rate of treatment was significantly better than that of calcipotriol, and the differences were statistically significant. In addition, the efficacy of defubao (1* *time/day) and calcipotriol (2* *times/day) was compared.

Five randomized controlled trials compared the effect of defubao and other drugs by comparing the baseline change rate of PASI before and after 8 weeks of treatment. Based on the provided clinical trial data, we conducted a descriptive analysis of the trial results, as shown in Figure 6.

### 4.2. Security Analysis

Six studies compared the safety issues of using defubao and calcipotriol. Three randomized experiments compared the safety difference of treatment for 4 weeks, and 3 randomized controlled experiments compared the safety difference of treatment for 8 weeks. Meta-analysis uses a fixed-effects model to compare the occurrence of adverse events. The results suggest that the defubao group was used for 4 weeks or 8 weeks. The incidence of adverse events was significantly less than that of the calcipotriol group. The funnel chart shows asymmetry, and there is a publication offset in the research, as shown in Figure 7.

Four randomized controlled trials compared the safety of defubao and betamethasone for 8 weeks of treatment, that is, the proportion of at least one adverse event. The results showed that after 8 weeks of treatment with defubao and betamethasone, there was no statistical difference in the incidence of adverse reactions between the two. Two randomized controlled trials compared the incidence of adverse reactions after using Defabao and placebo for 4 weeks. Through data analysis, it was found that the proportion of adverse events in the placebo group was significantly higher than that in the defubao group. The results of different groups for 8 weeks are shown in Figure 8. In addition, the safety analysis and comparison results are shown in Table 2.

### 4.3. Discussion

Relevant scholars observed the changes in clinical PASI score and vascular dilatation under dermatoscope after treatment, and the relative index was used to calculate the evaluation index [36]. Many published evaluation indicators for observing curative effect are compared with the decline rate. In the initial stage of the trial design, this article consulted a large number of domestic and foreign literatures and found that even if the psoriatic skin lesions appear normal to the naked eyes, the capillaries still have different degrees of expansion under dermoscopy [37]. With drug treatment, the skin lesions of psoriasis improved, and the improvement of skin lesions reduced the release of vascular growth factors and inflammatory mediators, which in turn changed the state of intravascular microcirculation of the whole body skin, and the intravascular microcirculation of the skin surrounding the skin lesions. It will change accordingly, that is, the “normal skin data around the skin lesion” will change. The comprehensive evaluation compared the relative index algorithm and the decline rate algorithm [38]. In this experiment, the decline rate was selected as the evaluation index, the target skin lesion score (TLS) was observed to evaluate the severity of the skin lesion, and the diameter of the vascular bulb was used to evaluate the degree of vasodilation, respectively.

In addition, in order to be able to observe the overall condition of the skin lesions under a dermatoscopic field of view, and reduce the error caused by the difference in the observation field, the area of the psoriasis skin lesions selected in this experiment is 4–9 cm^2^, which makes the data obtained more objective. However, this experiment only observed the changes in specific skin lesions of patients with psoriasis after treatment with defubao, and did not observe and evaluate the overall disease severity of the patients. In the study included in Study 1 (meta-analysis) of this article, it was found that the PASI score of patients with psoriasis vulgaris was significantly decreased after topical application of defubao. Because previous studies have found that in mouse experimental models, the inhibitory effect of steroid hormones on DNA synthesis can be observed even if they are far away from the site where steroid hormones are used [39]. In addition, the improvement of psoriasis plaques reduces the release of vascular growth factors and inflammatory mediators, and the intravascular microcirculation of the whole body skin will be improved.

The two main immunohistological changes in psoriasis are the changes in the skin microvascular system and the abnormal differentiation of the epidermis in the end-stage. The capillary loops in the dermal papilla can be seen elongated, bent and dilated. Relevant scholars have found that in the early stage of psoriasis, the skin lesions and surrounding capillaries dilate and abnormal blood flow precede the inflammatory manifestations and hyperplasia of the skin lesions [40]. With the treatment, the skin lesions improved, the plaque disappeared, and the degree of vasodilation and function also gradually recovered. The researchers compared the blood vessel diameters of scalp lesions in healthy people, patients with seborrheic dermatitis, and patients with psoriasis through dermoscopy, and found that the diameters of scalp capillaries in the seborrheic dermatitis group and the healthy group were similar [41]. There was a significant difference between the capillary diameter of the group and the former two, and the vascular bulb was significantly expanded. In recent years, the use of noninvasive examination methods to evaluate the efficacy of drugs has increasingly appeared in several skin diseases including psoriasis. After local or systemic drug treatment, the researchers evaluated the effect of the drug by evaluating the change in the diameter of the capillary globules in psoriasis or the number of capillary globules per unit field of view before and after the treatment [42].

This article compares the effectiveness and safety differences of defubao, calcipotriol, betamethasone, and placebo in the treatment of psoriasis vulgaris. Regardless of the treatment for 2 weeks, 4 weeks, or 8 weeks, compared with the calcipotriol group, the betamethasone group, or the placebo group, the efficacy of the defubao group was more significant. Topical calcipotriol and glucocorticoids are classic drugs for the treatment of psoriasis, but calcipotriol requires an alkaline environment to maintain stability, and betamethasone can be more effective in an acidic environment. The two are incompatible when mixed, and it is difficult to have both. For this reason, the researchers developed a unique and stable excipient to overcome the incompatibility barrier of the two, and finally form a formulation containing stable active ingredients. This not only gives play to the advantages of the two drugs, makes the treatment effect stronger, but also reduces the amount of topical glucocorticoids, thereby reducing the risk of hormone-related adverse reactions. This may be the reason why defubao is better than calcipotriol and betamethasone. In addition, meta-analysis found that after 4 weeks of treatment, the effective rate of the defubao group (1* *times/day) was 1.72 times that of the calcipotriol group (2* *times/day), which provides powerful clinical guidance for medication However, the low frequency of medication and the significant effect are more acceptable to patients. From the perspective of pharmacoeconomics, it can reduce costs and is more beneficial to patients. The study found that the incidence of adverse events in the calcipotriol group was significantly higher than that in the defubao group, while the difference in adverse events between the defubao group and the betamethasone group was not statistically significant. Moreover, it is mentioned in the literature that long-term use of defubao will not increase the risk of glucocorticoid-related adverse events compared with nonglucocorticoid topical drugs. This shows that the safety of defubao treatment is worthy of recognition.

This study found that within 8 weeks of medication, the curative effect increased with the time of medication, 8 weeks curative effect >4 weeks curative effect >2 weeks curative effect, and the difference between them was statistically significant. However, there is a lack of longer-term efficacy data. Therefore, clinical observations of a longer course of treatment are needed to determine the optimal medication time for treatment with defubao. This meta-analysis only compares the efficacy of defubao, calcipotriol and betamethasone, and does not compare with other topical drugs. This study included 11 studies, divided into multiple subgroups. When designing the study, the publication bias was tested by formulating detailed search strategies, searching literature from multiple libraries, formulating inclusion and exclusion criteria, sensitivity analysis, and making funnel charts. The number of studies included in some subgroups is small, which affects the results of heterogeneity testing. In addition, this study only retrieved Chinese and English articles, and did not retrieve research conclusions in other languages. All of the above may cause bias.

This study evaluated the efficacy of topical defubao on psoriasis vulgaris. Through clinical observation and dermoscopic observation, it was found that defubao had a significant effect on psoriasis skin lesions. The treated psoriasis plaques improved in all patients, and at the same time, the diameter of the capillary bulbs under dermoscopy gradually decreased.

However, there is a big difference between the speed and intensity of the improvement of the diameter of the capillary bulb under the dermoscopy and the clinical TLS score. After 4 weeks of treatment, the TLS score was 25/32 of “completely healed skin lesions” and “significantly improved”, which reached almost 78%, while the spheroid diameter score was much lower than 10%. After 6 weeks of treatment, the target skin lesions of 26 patients had completely disappeared. Under dermoscopic imaging observations, only 5 patients returned to normal vascular diameters, while in other patients, even those whose clinical skin lesions disappeared completely, there were still significant telangiectasias.

There may be two mechanisms for the difference in results between the two. One possibility is that we have observed that the psoriasis skin lesions have subsided clinically, but there may still be slight keratinocyte proliferation or low-level growth factor secretion in the skin lesions. These small changes may continue to stimulate blood vessel formation. Another possibility is that the regulation speed of the keratinocyte proliferation cycle is faster than the speed of capillary remodeling or disappearance, the proliferation cycle of keratinocytes has returned to normal, but the expanded capillaries still exist. After treatment, some psoriasis skin lesions have dilated capillaries that can become smaller, but they cannot return to their normal size. As we all know, all clinical treatment observations are performed with standard doses within the safe range of each drug, so it cannot be excluded that increasing the dose of the drug can improve the microcirculation changes of the psoriasis skin lesions and make it possible for the dilated blood vessels to return to normal.

This article not only searched the English database, but also searched the Chinese database. The included studies are more comprehensive and involve more ethnic groups. The comparisons were made with PASI, IGA, and PGA as evaluation indicators, and the results obtained were more comprehensive and objective. The included articles are all high-quality randomized controlled trials, divided into multiple subgroups, and stratified analysis of the difference in efficacy of 2 weeks, 4 weeks, and 8 weeks of treatment.

## 5. Conclusion

This paper studies the classic algorithm Apriori in association rules, points out the insufficiency of this algorithm and the existing improved algorithms in dealing with unbalanced medical data sets, and then proposes a new scheme of mining association rules after balancing first to improve it. A new scheme for mining association rules that balances first and then mines is proposed. In the data balance part, aiming at the blind sampling problem of the traditional SMOTE algorithm, a balance improvement algorithm based on the combination of K-means and SMOTE is proposed. Defubao was safer than calcipotriol and placebo. The difference was statistically significant, but there was no statistical difference from betamethasone. Defubao is more advantageous than calcipotriol or betamethasone in the treatment of psoriasis vulgaris. High-quality systematic reviews provide an effective and objective choice for the choice of clinical external medications. Two randomized controlled trials were conducted to compare the efficacy of defubao in the treatment of psoriasis vulgaris in 2, 4, and 8 weeks. A fixed-effect model was used for data analysis, and the results showed that the efficacy after 4 weeks of use was better than that after 2 weeks of use [OR = 0.73, 95% CI (0.61, 0.86), *P* < 0.01]. The curative effect after 8 weeks of use was significantly better than that after 4 weeks of use [OR = 0.68, 95% CI (0.47, 0.98), *P* < 0.01]. The curative effect after 2 weeks of use was significantly weaker than that after 8 weeks of use [OR = 0.49, 95% CI (0.41, 0.58), *P* < 0.01]. After topical treatment of psoriasis skin lesions with defubao, the clinical observation showed that the skin lesions subsided and the diameter of the vascular bulb became smaller under dermatoscope, suggesting that defubao is effective in treating psoriasis vulgaris. There is a positive correlation between the target skin lesion score of a specific skin lesion in psoriasis and the diameter of the vascular bulb. As the treatment time increases, the correlation between the two increases. The reduction rate of the clinical target skin lesion score after treatment of psoriasis skin lesions is significantly greater than the reduction rate of vascular globule diameter. The microvascular healing of the skin lesions is later than the clinical cure. The observation of skin lesion vascular changes can be used to evaluate the condition of psoriasis and guide drug selection. However, this study only compared the efficacy of defubao, calcipotriol and betamethasone, and did not compare with other topical drugs. Further research is needed. In addition, there is also a lack of data to study the longer-term efficacy of defubao.

## Figures and Tables

**Figure 1:** Apriori calculation process.

**Figure 2:** Architecture of psoriasis data mining system based on association rules.

**Figure 3:** Random forest algorithm process.

**Figure 4:** IGA as an indicator to evaluate the 8-week defubao group and the betamethasone group.

**Figure 5:** IGA was used to evaluate the 8-week defubao group and the calcipotriol group.

**Figure 6:** PASI reduction rate for 8 weeks of treatment.

**Figure 7:** Safety analysis of the 8-week defubao group and the calcipotriol group.

**Figure 8:** Safety analysis results of different groups in 8 weeks.

**Table 1:** Transaction matrix D1.

	I1	I2	I3	I4	I5
T1	1	2	1	2	1
T2	2	1	1	1	2
T3	2	1	1	2	1
T4	1	2	2	1	2
T5	1	2	2	1	1

**Table 2:** Comparison results of safety analysis.

Outcome indicators	*χ* ^2^	Heterogeneity p	OR	0.95CI	Z	*P*
Defubao vs placebo 4 weeks	0.01	0.52	0.61	(0.41,0.89)	2.3	0.02
Defubao vs betamethasone 8 weeks	0	0.93	0.92	(0.84,1.1)	0.56	0.16
Defubao vs calcipotriol 8 weeks	0.65	0.03	0.57	(0.48,0.66)	6.4	0.011
Defubao vs calcipotriol 4 weeks	0.32	0.21	0.52	(0.42,0.61)	5.2	0

## Data Availability

Relevant data require the consent of the corresponding author to obtain it.
